# MicroRNA-98 acts as a tumor suppressor in hepatocellular carcinoma via targeting SALL4

**DOI:** 10.18632/oncotarget.12190

**Published:** 2016-09-22

**Authors:** Wuyuan Zhou, Benkui Zou, Lisheng Liu, Kai Cui, Jie Gao, Shuanghu Yuan, Ning Cong

**Affiliations:** ^1^ Department of Hepatobillary Surgery, Shandong Cancer Hospital, Jinan, Shandong 250117, P.R. China; ^2^ Department of Urology Surgery, Shandong Cancer Hospital, Jinan, Shandong 250117, P.R. China; ^3^ Clinical Laboratory, Shandong Cancer Hospital, Jinan, Shandong 250117, P.R. China; ^4^ Department of Radiation Oncology, Shandong Cancer Hospital, Jinan, Shandong 250117, P.R. China; ^5^ Department of Intervention Therapy, Shandong Cancer Hospital, Jinan, Shandong 250117, P.R. China

**Keywords:** hepatocellular carcinoma, microRNA-98, tumor suppressor, SALL4

## Abstract

MicroRNAs (miRs) are involved in the development and progression of hepatocellular carcinoma (HCC), but the regulatory mechanism of miR-98 in HCC still remains unclear. Here we found that miR-98 was significantly downregulated in HCC tissues compared to matched adjacent normal tissues (ANTs). Low miR-98 expression was associated with tumor size, metastasis, portal vein tumor embolus, and poor overall survival. Ectopic expression of miR-98 decreased the proliferation, migration, invasion and epithelial-mesenchymal transition (EMT) of HCC cells. SALL4 was identified as a novel target of miR-98, and the protein expression of SALL4 was inhibited by miR-98 in HCC cells. Overexpression of SALL4 reversed the suppressive effects of miR-98 on the malignant phenotypes of HCC cells. Besides, SALL4, upregulated in HCC tissues compared to the matched ANTs, was inversely correlated to the miR-98 levels in HCC tissues. In addition, overexpression of miR-98 markedly suppressed the tumor growth as well as tumor-induced death in nude mice. In summary, miR-98 plays a suppressive role in the proliferation, migration, invasion and EMT of HCC cells, partly at least, via directly inhibition of SALL4. Therefore, the miR-98/SALL4 axis may become a promising therapeutic target for HCC.

## INTRODUCTION

Hepatocellular carcinoma (HCC), one of the most common cancers in human, causes 1 million deaths a year, and thus is one of the leading causes of cancer-related death worldwide [1, 2]. Understanding of the molecular mechanisms underlying HCC is important for the development of effective treatment strategies, and deregulations of oncogenes or tumor suppressors have been demonstrated to be involved in the development and progression of HCC [3, 4].

MicroRNAs (miRs), a kind of short non-coding RNAs, can induce mRNA degradation or translation inhibition through directly binding to the 3′-untranslational region (UTR) of their target genes [5]. Many miRs have been reported to participate in the regulation of a variety of biological processes, such as cell proliferation, differentiation, apoptosis, cell cycle progression, migration, and tumorigenesis [6–8]. Moreover, deregulations of miRs are implicated in the development and malignant progression of human cancers via inhibition of their targets that are oncogenes or tumor suppressors [9, 10]. Recently, deregulations of many miRs have been implicated in the growth and metastasis of HCC, such as miR-21 [11], miR-101 [12], miR-124 [13], miR-203 [13], and miR-148 [14], which may be used as potential therapeutic targets or candidates for HCC treatment.

MiR-98, belongs to the let-7/miR-98 family, acts as an oncogene or tumor suppressor in some human cancers through inhibiting the protein expression of its different target genes [15, 16]. For instance, miR-98 could suppress the growth and metastasis of oral squamous cell carcinoma by inhibiting the expression of IGF1R [17]. Ni et al. reported that miR-98 targeted ITGB3 to inhibit proliferation, migration, and invasion of non-small-cell lung cancer [18]. Li et al. showed that miR-98 inhibited melanoma metastasis through a negative feedback loop with its target gene IL-6 [19]. Recently, Lin-28B, a RNA-binding protein, was suggested to promote tumor formation and invasion in HCC through coordinated repression of the let-7/miR-98 family and induction of multiple oncogenic pathways [20]. However, the exact role of miR-98 in the progression of HCC as well as the underlying mechanism still remains to be fully uncovered.

Sal-like protein 4 (SALL4) is a zinc finger transcription factor, and has recently been identified as a marker for stem cells, involved in the maintenance of self-renewal in embryonic stem cells [21]. Moreover, SALL4 was found to be mainly expressed in fetal livers, and was identified as an important biomarker for several common human cancers [22, 23]. Upregulation of SALL4 is found in HCC, breast cancer and endometrial cancer, predicting a poor prognosis [24–26]. Furthermore, SALL4 could promote the tumorigenesis and malignant progression of HCC [27–29]. Therefore, SALL4 may become a promising molecular target for the treatment of HCC. However, till to now, the regulatory mechanism of SALL4 in HCC remains largely unknown.

In this study, we aimed to investigate the regulatory mechanism of miR-98 in the progression of HCC.

## RESULTS

### MiR-98 is downregulated in HCC

To reveal the role of miR-98 in HCC, real-time RT-PCR was performed to examine the miR-98 levels in a total of 144 HCC tissues and ANTs. As shown in Figure 1A, the miR-98 levels were indeed significantly decreased in HCC tissues compared to ANTs. We then investigated the association between the miR-98 expression and the clinicopathological features of HCC. All HCC patients involved in this study were divided into high miR-98 expression group and low miR-98 expression group, according to the mean value of the miR-98 level as the cutoff point. As indicated in Table 1, 88 cases (61.1%) were in the low miR-98 level group, while 56 cases (38.9%) were in high miR-98 level group. Moreover, the decreased miR-98 levels were significantly associated with tumor size, metastasis, and portal vein tumor embolus (Table 1). However, no statistically significant association of miR-98 expression was found with the age, gender, AFP, HBV infection, or cirrhosis (Table 1). These findings suggest that downregulation of miR-98 may contribute to the malignant progression of HCC.

**Figure 1:** MiR-98 is downregulated in HCC, associated with malignant progression and poor prognosis **A.** Real-time qPCR was conducted to determine the miR-98 levels in a total of 144 primary HCC tissues and matched adjacent normal tissues (ANTs). Data are represented as mean +/− SD. ** means P<0.01 vs. ANTs. **B.** Survival analysis indicated that the HCC patients with low miR-98 levels had shorter survival time compared with those with high miR-98 levels.

**Table 1:** Association between miR-98 expression and clinicopathologic features of patients with hepatocellular carcinoma

Variables	Number	Low miR-98 (n=88)	High miR-98 (n=56)	P value
**Age**				
<55	56	35	21	0.86
≥55	88	53	35	
**Gender**				
Male	84	52	32	0.86
Female	60	36	24	
**Tumor size**				
<5 cm	86	46	40	0.025*
≥5 cm	58	42	16	
**Metastasis**				
No	66	33	33	0.016*
Yes	78	55	23	
**Portal vein tumor embolus**				
No	73	38	35	0.027*
Yes	71	50	21	
**AFP**				
Negative	75	47	28	0.73
Positive	69	41	28	
**HBV infection**				
No	39	22	17	0.56
Yes	105	66	39	
**Cirrhosis**				
No	74	43	31	0.5
Yes	70	45	25	

* means the difference has statistical significance.

We further performed overall survival analysis (Kaplan-Meier analysis) for these HCC patients. As indicated in Figure 1B, the HCC patients with low miR-98 levels had shorter survival time when compared with those with high miR-98 levels, which further suggests that downregulation of miR-98 may predicate poor prognosis of HCC patients.

### MiR-98 inhibits proliferation, migration, invasion and EMT of HCC cells

To further study the regulatory role of miR-98 in HCC, two common HCC cell lines HepG2 and SMMC-7721 were transfected with miR-98 mimic to upregulate its expression. Real-time RT-PCR data indicated that the miR-98 level was significantly increased in the miR-98 group compared to the control group without any transfection (Figure 2A and 2B). MTT assay was then conducted to determine the cell proliferation. As shown in Figure 2C and 2D, overexpression of miR-98 significantly decreased the proliferation of HepG2 and SMMC-7721 cells. After that, wound healing assay and transwell assay were performed to examine the cell migration and invasion, respectively. Our data showed that the cell migration and invasion were downregulated in the miR-98 group compared to the control group (Figure 3A-3D).

**Figure 2:** MiR-98 suppresses HCC cell proliferation HCC HepG2 and SMMC-7721 cells transfected with miR-98 mimic or scramble miR mimic (miR-NC). Non-transfected HepG2 and SMMC-7721 cells were used as controls. **A, B.** Real-time RT-PCR was conducted to determine the miR-98 expression. **C, D.** MTT assay was performed to determine cell proliferation. Data are represented as mean +/− SD. ** means P<0.01 vs. HepG2 or SMMC-7721.

**Figure 3:** MiR-98 inhibits migration and invasion of HCC cells HCC HepG2 and SMMC-7721 cells transfected with miR-98 mimic or scramble miR mimic (miR-NC). Non-transfected HepG2 and SMMC-7721 cells were used as controls. **A, B.** Wound healing assay and **C, D.** transwell assay were performed to determine cell migration and invasion Data are represented as mean +/− SD. ** means P<0.01 vs. HepG2 or SMMC-7721. (400x for transwell assay, 40x for wound healing assay).

In addition, MMP2 and MMP9, two key matrix metalloproteinases involved in tumor cell migration and invasion, were also downregulated after miR-98 overexpression in HepG2 and SMMC-7721 cells (Figure 4A-4B). We further examined the protein levels of epithelial-mesenchymal transition (EMT)-related factors. Western blot data indicated that that after miR-98 upregulation, the E-cadherin protein levels were increased, while the protein levels of N-cadherin, Fibronectin, vimentin were reduced in HepG2 and SMMC-7721 cells (Figure 4C-4D), indicating that the EMT is downregulated after overexpression of miR-98 in HCC cells. Accordingly, miR-98 plays a suppressive role in the regulation of cell proliferation, migration, invasion and EMT of HCC cells.

**Figure 4:** MiR-98 inhibits MMPs expression and epithelial-mesenchymal transition (EMT) in HCC cells HCC HepG2 and SMMC-7721 cells transfected with miR-98 mimic or scramble miR mimic (miR-NC). Non-transfected HepG2 and SMMC-7721 cells were used as controls. **A, B.** Western blot was used to examine the protein levels of MMP2/9. **C, D.** Western blot was used to examine the protein levels of EMT-related genes. Data are represented as mean +/− SD. ** means P<0.01 vs. HepG2 or SMMC-7721.

### SALL4 is a direct target gene of miR-98 in HCC cells

We then used TargetScan, PicTar, and miRanda to analyze the potential targets of miR-98. As indicated in Figure 5A, SALL4 was a putative target gene of miR-98, and perfect base pairing was observed between the seed sequence of mature miR-98 and the 3′UTR of SALL4. To verify this predication, we subcloned the WT or MT of SALL4 3′UTR into a luciferase reporter vector, respectively (Figure 5B). Luciferase reporter assay was then conducted. As indicated in Figure 3C, co-transfection with WT-SALL4-3′UTR plasmid and miR-98 mimic led to a significant decrease in the luciferase activity. However, co-transfection with MT-SALL4-3′UTR plasmid and miR-98 mimic had not effect on the luciferase activity (Figure 5C and 5D). These findings indicate that miR-98 can directly bind to seed sequence in the 3′UTR of SALL4.

**Figure 5:** SALL4 is a target gene of miR-98 in HCC cells **A.** The seed sequences of miR-98 in the wild type and mutant type 3′UTR of SALL4 are indicated. **B.** Representation of the vectors containing the wild type (WT) or mutant type (MT) 3′UTR of SALL4 used in the Luciferase assay. **C, D.** The luciferase activity was notably decreased in HCC HepG2 and SMMC-7721 cells co-transfected with miR-98 mimics and WT-SALL4-3′UTR reporter plasmid, but unaltered in HepG2 and SMMC-7721 cells co-transfected with miR-98 mimics and MT-SALL4-3′UTR plasmid. **E, F.** Western blot was conducted to examine the protein expression of SALL4 in HepG2 and SMMC-7721 cells transfected with miR-98 mimic or scramble miR mimic. Non-transfected HepG2 and SMMC-7721 cells were used as controls. Data are represented as mean +/− SD. ** means P<0.01 vs. HepG2 or SMMC-7721.

As miRs could inhibit the translation of their target genes [7], we further conducted western blot to examine the protein level of SALL4 in HepG2 and SMMC-7721 cells after overexpression of miR-98. We found that the protein expression of SALL4 was significantly decreased in the miR-98 group compared to the miR-NC group (Figure 5E and 5F). Taken together, our data demonstrate that miR-98 can inhibit the protein expression of SALL4 via binding to the 3′UTR of SALL4 in HCC cells.

### Overexpression of SALL4 reverses the suppressive effects of miR-98 on HCC cells

As SALL4 has been found to be an important oncogene in HCC [30], we speculated that SALL4 might be involved in miR-98-mediated inhibition of the malignant phenotypes of HCC cells. To clarify this speculation, we performed the reverse experiments. MiR-98-overexpressing HepG2 and SMMC-7721 cells were further transfected with pcDNA3.1-SALL4 plasmid to restore its expression. After transfection, western blot data showed that the decreased SALL4 level was significantly upregulated (Figure 6A-6B). MTT assay, wound healing assay and transwell assay were then conducted to examine the cell proliferation, migration and invasion, respectively. As demonstrated in Figure 6C-6D, the cell proliferation was significantly increased in the miR-98+SALL4 group, when compared with those in the miR-98 group. Similarly, the migration and invasion capacities of HCC cells were also higher in the miR-98+SALL4 group, when compared with those in the miR-98 group, respectively (Figure 7A-7D).

**Figure 6:** Overexpression of SALL4 attenuates the suppressive effects of miR-98 on HCC cell proliferation HepG2 and SMMC-7721 cells were transfected with miR-98 mimic, or co-transfected with miR-98 mimic and SALL4 plasmid, respectively. **A, B.** Western blot was conducted to examine the protein expression of SALL4. **C, D.** MTT assay were performed to examine cell proliferation. Data are represented as mean +/− SD. ** means P<0.01 vs. miR-98.

**Figure 7:** Overexpression of SALL4 eliminates the inhibitory effects of miR-98 on HCC cell migration and invasion HepG2 and SMMC-7721 cells were transfected with miR-98 mimic, or co-transfected with miR-98 mimic and SALL4 plasmid, respectively. **A, B.** Wound healing assay and **C, D.** transwell assay were performed to determine cell migration and invasion, respectively. Data are represented as mean +/− SD. ** means P<0.01 vs. miR-98. (400x for transwell assay, 40x for wound healing assay).

The protein levels of invasion- and EMT-related proteins were then determined using western blot. Consistent with the transwell assay data, the MMP2 and MMP9 protein levels were significantly increased in the miR-98+SALL4 group compared to the miR-98 group (Figure 8A-8B). Besides, the E-cadherin protein levels were reduced, while the Fibronectin, N-cadherin and vimentin protein levels were increased in the miR-98+SALL4 group compared to the miR-98 group (Figure 8C-8D), suggesting that the EMT was promoted after restoration of SALL4 expression in HCC cells. Accordingly, our data demonstrate that overexpression of SALL4 reversed the inhibitory effects of miR-98 on the malignant phenotypes of HCC cells, suggesting that the suppressive role of miR-98 in HCC is through inhibition of SALL4.

**Figure 8:** Overexpression of SALL4 eliminates the inhibitory effects of miR-98 on MMPs expression and EMT in HCC cells HepG2 and SMMC-7721 cells were transfected with miR-98 mimic, or co-transfected with miR-98 mimic and SALL4 plasmid, respectively. **A, B.** Western blot was used to examine the protein levels of MMP2/9. **C, D.** Western blot was used to examine the protein levels of EMT-related genes. Data are represented as mean +/− SD. ** means P<0.01 vs. miR-98.

### SALL4 is reversely correlated with miR-98 in HCC

SALL4 has previously been demonstrated to be upregulated in HCC tissues and act as an important oncogene in HCC [30]. As we found that SALL4 was a direct target gene of miR-98, and was involved in the miR-98-mediated malignant phenotypes in HCC *in vitro*, we speculated that the downregulation of miR-98 might contribute to the upregulation of SALL4 in HCC tissues. To verify this speculation, we then conducted real-time RT-PCR to examine the SALL4 expression in HCC tissues and ANTs, and analyzed the correlation between the miR-98 and SALL4 levels in HCC tissues. Real-time RT-PCR data indicated that SALL4 was indeed upregulated in HCC tissues compared to ANTs (Figure 9A). Moreover, we found that the SALL4 levels were reversely correlated to the miR-98 levels in HCC tissues (Figure 9B). These findings suggest that the upregulation of SALL4 may be caused by the downregulation of miR-98 in HCC.

**Figure 9:** SALL4 is upregulated in HCC and inversely correlated to miR-98 levels **A.** Real-time qPCR was conducted to determine the mRNA levels of SALL4 in a total of 144 primary HCC tissues and matched adjacent normal tissues (ANTs). Data are represented as mean +/− SD. ** means P<0.01 vs. ANTs. **B.** An inverse correlation was observed between the miR-98 and SALL4 mRNA levels in HCC tissues.

### MiR-98 inhibits the growth of HCC *in vivo*

Finally, the effect of miR-98 on HCC growth *in vivo* was studied. MiR-98 was cloned into the pLVX-IRES-ZsGreen1 lentiviral vector, generating the pYr-LVX-miR-98 plasmid, which was stably transfected into HepG2 cells. While in the control group, HepG2 cells were stably transfected with the blank pLVX-IRES-ZsGreen1 vector. Real-time RT-PCR data showed that the miR-98 level was significantly upregulated in the miR-98 group, when compared to the control group (Figure 10A). After that, nude mice were subcutaneously implanted with HepG2 cells stably overexpressing miR-98. The tumor of HCC cells grew gradually after implantation. In the control group, all 5 mice died from the 53th to the 65th days after implantation; however, only 1 mouse died in the miR-98 group, indicating that overexpression of miR-98 protected nude mice from death caused by overexpression of miR-98 in HepG2 cells (Figure 10B). On the 65^th^ day after implantation, all mice if not died were sacrificed. As indicated in Figure 10C, the HCC xenograft was obtained, and the tumor was smaller in the miR-98 group compared to the control group. Moreover, the tumor volume and weight were significantly lower in the miR-98 group, when compared with those in the control group (Figure 10D-10E).

**Figure 10:** **A.** HepG2 cells were stably transfected with the blank pLVX-IRES-ZsGreen1 vector as Control or pYr-LVX-miR-98 lentiviral plasmid, and real-time RT-PCR was conducted to examine the miR-98 level in each group. **B.** Nude mice were subcutaneously implanted with HepG2 cells stably transfected with pYr-LVX-miR-98 lentiviral plasmid or blank pLVX-IRES-ZsGreen1 vector, respectively. The survival curve was indicated. **C.** On 65 days after implantation, the nude mice in each group were sacrificed, and the HCC xenograft was obtained. **D, E.** The tumor volume and weight were calculated. Data are represented as mean +/− SD. ** means P<0.01 vs. Control.

## DISCUSSION

Deregulations of MiR-98 participate in the development and progression of some cancers [15, 19]. Some studies have demonstrated that miR-98 has suppressive effects on oral squamous cell carcinoma [17], non-small-cell lung cancer [18], glioma [31], and melanoma [19], and plays an inhibitory role in tumor angiogenesis and invasion by inhibition of ALK4 and MMP11 [32]. On the contrary, however, miR-98 was also found to be significantly upregulated in gastric cancer [33], colon cancer [34], and small-cell lung cancer [35], and inhibited the expression of tumor suppressor gene FUS1 [35]. Pathak et al. found that the upregulated miR-98 was associated with colon cancer pathways and correlated with cyto- or chemokine expression [34]. Thus, the cancer-specific miR-98 may exert anti-tumor or oncogenic effects, depending on the cancer type. Here we found that the miR-98 levels were significantly reduced in HCC tissues compared to ANTs. Moreover, low miR-98 expression was significantly associated with the tumor size, metastasis, portal vein tumor embolus, and poor overall survival, suggesting that downregulation of miR-98 is involved in the HCC progression, and miR-98 may become a potential predicator for the prognosis of patients with HCC.

As miR-98 was downregulated in HCC, we transfected HepG2 and SMMC-7721 cells with miR-98 mimic to upregulate its expression. Restoration of miR-98 significantly suppressed the proliferation, migration and invasion of HepG2 and SMMC-7721 cell lines, suggesting that it may have inhibitory effect on HCC growth and metastasis. Similar findings were also shown in oral squamous cell carcinoma [17], non-small-cell lung cancer [18], glioma [31], and melanoma [19].

Cancer cells of epithelial origin can metastasize by transforming into cells with a mesenchymal phenotype, which is called EMT [36, 37]. During EMT, epithelial cells gradually lose their connection to the basement membrane, with increased invasive potential, and can degrade the extracellular matrix [36, 37]. Moreover, EMT is also characterized by the decreased expression of cell adhesion molecules such as E-cadherin, transformation of cytokeratin into vimentin, and alteration into the mesenchymal cell morphology [36, 37]. Therefore, EMT is very important for cancer cell migration and invasion [37]. In this study, overexpression of miR-98 significantly increased the expression of E-cadherin, while reduced the protein levels of N-cadherin, fibronectin and vimentin, indicating that EMT was inhibited. These findings were consistent with the migration and invasion data.

We further identified SALL4 as a novel target gene of miR-98, and found that miR-98 could inhibit the protein expression of SALL4 in HCC cells. SALL4 is an oncofetal protein that is expressed in the human fetal liver and silenced in the adult liver, but it is reexpressed in HCC patients, and high SALL4 level was associated with an unfavorable prognosis of patients with HCC [29, 30]. In addition, SALL4 promoted the proliferation, invasion, migration, EMT, chemoresistance, and the maintenance of cancer stem cells in different cancer types, and targeted inhibition of SALL4 has shown efficient therapeutic effects on cancer [22, 28, 38–40]. For instance, knockdown of SALL4 causes inhibition of lung cancer cell proliferation, induced by cell cycle arrest at the G1/early S phase [41]. In the present study, we found that restoration of SALL4 reversed the suppressive effect of miR-98 on the proliferation, migration, invasion and EMT of HCC cells, suggesting that miR-98 plays a suppressive role in HCC via inhibition of SALL4. To further confirm these findings, we examined the SALL4 expression in HCC tissues, and found that the SALL4 levels were reversely correlated with miR-98, supporting that downregulation of miR-98 may contribute to the upregulation of SALL4 in HCC. *In vivo* study further showed that overexpression of miR-98 significantly inhibited the tumor growth of HCC cells in nude mice, and protected them from tumor-induced death. These findings further suggest that miR-98 inhibits the HCC growth by inhibition of SALL4.

In summary, we reveals a tumor suppressive role of miR-98 in HCC, partly at least, via inhibition of SALL4, suggesting that the miR-98/SALL4 axis may become a promising therapeutic target for HCC treatment. The limitations of this study are that the number of HCC patients is only 144, not very large, and their clinical information is not comprehensive enough. Future studies should further investigate the upstream regulatory mechanism underlying miR-98 expression as well as the downstream signaling pathways of SALL4 in HCC cells, which may help expand the understanding of miR-98/SALL4 axis in HCC.

## MATERIALS AND METHODS

### Ethics statement

The study was approved by the Ethics Committee of Shandong Cancer Hospital, Jinan, China, and written informed consents were obtained from all studied patients.

### Clinical specimens

A total of 144 cases of HCC tissue specimens and matched adjacent normal tissues (ANTs) were obtained from Shandong Cancer Hospital between January 2012 and January 2013. All specimens had been confirmed by pathologists in our hospital. The clinicopathological information of these patients was summarized in Table 1. Patients involved in this study received neither radiation therapy nor chemotherapy before surgical resection. All tissue samples were immediately snap-frozen in liquid nitrogen after surgical resection and stored at −80°C until use.

### Cell lines

Human HCC cell lines HepG2 and SMMC-7721 were purchased from the Chinese Academy of Sciences (Shanghai, China). Cells were cultured in Dulbecco's modified Eagle's medium (DMEM, Life Technologies) supplemented with 10% fetal bovine serum (FBS, Life Technologies), 100 IU/ml penicillin and 100 IU/ml streptomycin. Cells were cultured at 37°C in a humidified atmosphere with 5% CO_2_.

### Real-time RT-PCR assay

Total RNA was extracted by using Trizol Reagent (Life Technologies). For miRs detection, a MiRNA Reverse Transcription Kit (Life Technologies) was used to convert RNA into cDNA, according to the manufacture's instruction. Real-time PCR was then performed by using a miRNA Q-PCR Detection Kit (GeneCopoeia, Rockville, MD, USA) on ABI 7500 thermocycler. U6 gene was used as an internal reference. For mRNA detection, Reverse Transcription Kit (Life Technologies) was used to convert RNA into cDNA, according to the manufacture's instruction. Real-time PCR was then performed by using Q-PCR Detection Kit (Life Technologies) on ABI 7500 thermocycler. The sequences of primers for SALL4, Forward: 5′-CCAGGGAATGACGAGGTGG-3′; Reverse: 5′-GAACTCCGCACAGCATTTCTC-3′. The sequences of primers for GAPDH, Forward: 5′- GGAGCGAGATCCCTCCAAAAT-3′; Reverse: 5′- GGCTGTTGTCATACTTCTCATGG-3′. The PCR steps were 95°C for 10 min, and 40 cycles of denaturation at 95°C for 15 sec and annealing/elongation step at 60°C for 60 sec. The relative miR-98 expression was normalized to U6. The relative expression was analyzed by the 2^−ΔΔCt^ method [42].

### Western blot

Cells were lysed with ice-cold lysis buffer (50 mM Tris-HCl, pH 6.8, 100 mM 2-ME, 2 %w/v SDS, 10 % glycerol). After centrifugation at 20,000×g for 10 min at 4 °C, proteins in the supernatants were quantified and separated with 10% SDS-PAGE. Then, proteins were transferred onto a polyvinylidene difluoride (PVDF) membrane (Amersham Bioscience, Buckinghamshire, USA), which was then incubated with PBS containing 5% milk overnight at 4 °C. The PVDF membrane was incubated with rabbit anti-human primary antibodies including SALL4 (polyclonal, 1:100, ab29112), E-cadherin (polyclonal, 1:50, ab15148), N-cadherin (polyclonal, 1:50, ab18203), Fibronectin (polyclonal, 1:200, ab2413), vimentin (monoclonal, 1:50, ab16700), MMP2 (polyclonal, 1:200, ab37150), MMP9 (polyclonal, 1:100, ab38898), and GAPDH (polyclonal, 1:100, ab181602) (all from Abcam, Cambridge, MA, USA) at room temperature for 3 h, respectively, and then with mouse anti-rabbit secondary antibody (monoclonal, 1:10000, ab99702, Abcam) at room temperature for 1 h. Super Signal West Pico Chemiluminescent Substrate Kit (Pierce, Rockford, IL, USA) was then used to detect signals, according to the manufacture's instruction. The relative protein expression was analyzed by Image-Pro plus software 6.0, represented as the density ratio versus GAPDH.

### Plasmid constructions

The full-length 3′-untranslated region (UTR) of SALL4 was amplified from human genomic DNA, and then cloned into the downstream of the firefly luciferase coding region of pMIR-GLOTM Luciferase vector (Promega, USA), named as pMIR-SALL4. Mutations of miR-98 binding sites were introduced by site-directed mutagenesis, which was then cloned into the downstream of the firefly luciferase coding region of pMIR-GLOTM Luciferase vector, named pMIR-Mut SALL4.

### Small interfering RNAs, miR mimic and inhibitor

The pcDNA3.1-SALL4 plasmid, miR-98 mimic, scramble miR mimic, were purchased from Amspring (Changsha, China).

### MTT assay

The 3-(4,5-dimethylthiazal-2-yl)-2,5-diphenyl-tetrazolium bromide (MTT) assay was used to examine cell proliferation [43]. Briefly, cells in each group were plated at a density of 10000 cells per well in 96-well plates. After cultured for 12, 24, 48 and 72 h, the cells were incubated with MTT at a final concentration of 0.5 mg/ml for 4 h at 37°C. After the removal of the medium, 150 mM DMSO solutions were added to dissolve the formazan crystals. The absorbance was read at 570 nm using a Bio-Tek™ ELX-800™ Absorbance Microplate reader.

### Cell migration assay

Wound healing assay was performed to evaluate the cell migratory capacity of HCC cells in each group. In brief, cells were cultured to full confluence. Wounds of approximately 1 mm width were created with a plastic scriber, and cells were washed and incubated in a serum-free medium. After wounding for 24h, cells were incubated in a medium including 10% FBS. After cultured for 48 h, cells were fixed and observed under a microscope (Olympus, Tokyo, Japan).

### Cell invasion assay

Cell invasion assay was performed using transwell chambers (BD, USA), which were pre-coated with Matrigel. Cell suspension containing 5×10^5^ cells/ml was prepared in serum-free media, and 300μl of cell suspension was added into the upper chamber. Then, 500 μl of DMEM with 10% FBS was added into the lower chamber. Cells were incubated for 24 h. Then, we used a cotton-tipped swab to carefully wipe out the cells that did not invade through the pores. The filters were fixed in 90 % alcohol and stained by crystal violet, and observed under an inverted microscope (Olympus, Tokyo, Japan).

### Luciferase reporter gene assay

Cells were seeded into 24-well plates and co-transfected with 200 ng of pMIR-SALL4 or pMIR-SALL4-Mut vector and 100 ng of miR-98 mimic or scramble miR mimic, and the pRL-TK plasmid (Promega, Madison, WI) as internal normalization. Cells were harvested after 36 h and lysed using the lysis buffer (Promega). Luciferase reporter gene assay was conducted by using the Dual-Luciferase Reporter Assay System (Promega), in accordance with the manufacturer's instruction.

### Stable transfection and tumor growth analysis

Male BALB/C-nu/nu nude mice (8 weeks) were purchased from the Animal Center of Central South University (Changsha, China), and maintained under specific pathogen-free condition at the Laboratory Animal Room of Shandong Cancer Hospital. The miR-98 was cloned into the pLVX-IRES-ZsGreen1 vector (Amspring) to construct the pYr-LVX-miR-98 lentiviral plasmid. HepG2 cells were then stably transfected with pYr-LVX-miR-98 lentiviral plasmid or blank pLVX-IRES-ZsGreen1 vector as controls. To determine the effect of miR-98 on the tumorigenesis of HCC cells *in vivo*, nude mice were injected subcutaneously in the dorsal flank with 5×10^6^ HepG2 cells stably transfected with miR-98-overexpressing plasmid. Besides, in the control group, nude mice were injected with 5×10^6^ HepG2 cells stably transfected with the blank vector. Survival time was recorded. Nude mice were sacrificed, if not died, on 65 days after tumor implantation. Tumor volume was calculated by using the formula V (mm^3^) = 0.5×a×b2 (a maximum length to diameter, b maximum transverse diameter). Tumor weight was also recorded when mice died.

### Statistical analysis

Data were expressed as mean ± standard deviation from at least three separate experiments. SPSS19.0 was used to perform statistical analysis. Qualitative data were analyzed by the chi-square test. Correlation was determined by Pearson correlation analysis. Independent t-tests were used to compare the differences between two groups. One-way ANOVA with Bonferroni post-hoc tests were performed to compare the differences among more than two groups. P<0.05 were considered statistically significant.
